The article "Detoxification II Prescription Suppresses the Th-17/IL-17 Inflammatory Axis to Improve the Liver Function of ACLF-Rats via Inactivating the P38MAPK Pathway" was published in 2021. Journal: J Healthc Eng.

# Detoxification II Prescription Suppresses the Th-17/IL-17 Inflammatory Axis to Improve the Liver Function of ACLF-Rats via Inactivating the P38MAPK Pathway

**DOI:** 10.1155/2021/7563383

**Published:** 2021-12-03

**Authors:** Qinglan Shi, Wenjie Bai, Dewen Mao, Yueqiao Chen, Kejing Wang, Hua Qiu, Jinyu Wu

**Affiliations:** ^1^Department of Liver Diseases, The First Affiliated Hospital of Guangxi University of Chinese Medicine, Nanning 530023, Guangxi Zhuang Autonomous Region, China; ^2^Department of Foreign Language, Guangxi University of Chinese Medicine, Nanning 530001, Guangxi Zhuang Autonomous Region, China; ^3^Hepatobiliary Surgical Department, Ruikang Hospital of Guangxi University of Chinese, Nanning 530011, Guangxi Zhuang Autonomous Region, China; ^4^Department of Rheumatism and Immunology, The First Affiliated Hospital of Guangxi University of Chinese Medicine, Nanning 530023, Guangxi Zhuang Autonomous Region, China

## Abstract

Hepatitis is a metabolic system disease which is a serious challenge to the medical and healthcare system of the world. This study attempted to investigate the therapeutic effect and illustrate the regulation pharmacological mechanism of Detoxification II Prescription on ACLF. In this study, the rats were injected with D-galactosamine to establish ACLF-rat models, and the levels of cholinesterase (CHE), alanine aminotransferase (ALT), aspartate aminotransferase (AST), albumin (ALB), and total bilirubin (TBiL) were measured with the related kits to reflect the liver functions of the rats. The levels of IL-17, IL-6, and IFN-*γ* in the serums of the rats were detected by qRT-PCR, and the percentages of Th-17 cells in CD4^+^ cells of the rats were measured by flow cytometry assay. In the results, the increased ALT, AST, TBiL, IL-6, IL-17, IFN-*γ*, and percentage of Th-17 cells in CD4^+^ and decreased ALB and CHE were found in the serums of the ACLF-rats, while Detoxification II Prescription could partly reverse those indexes of the ACLF-rats. Moreover, it was also found that Detoxification II Prescription could inhibit the expression of P38MAPK, and P38MAPK downregulation obviously improved the liver function indexes of the ACLF-rats including the levels of ALT, AST, TBiL, IL-6, IL-17, IFN-*γ*, and percentage of Th-17 cells in CD4^+^ cells. In conclusion, this study suggested that Detoxification II Prescription could suppress the Th-17/IL-17 inflammatory axis to improve the liver function of ACLF-rats via inhibiting the activity of the P38MAPK pathway.

## 1. Introduction

The liver plays a crucial role in the metabolic activities of human bodies, and the inflammation induced by metabolic burden, toxic substances, and some viruses may aggravate the injury of the liver and further mediate the organ dysfunction [1, 2]. Recently, ACLF has been focused on by many studies. The study has showed that the acute-on-chronic liver failure (ACLF) is one of the serious liver-related diseases with high mortality [3]. Statistically, the short-term mortality of the patients with ACLF is more than 50%, and the incidence of the ACLF is increasing year by year [4]. At present, liver transplantation is a major method in clinic for ACLF treatment, while the shortages of donor livers limit the efficiency of the treatment for the patients [5, 6]. Thus, more therapeutic strategies are necessary to counter this dilemma in the clinical treatment of ACLF.

The article "Detoxification II Prescription Suppresses the Th-17/IL-17 Inflammatory Axis to Improve the Liver Function of ACLF-Rats via Inactivating the P38MAPK Pathway" was published in 2021. Journal: J Healthc Eng.

In recent ten years, the clinical values of traditional Chinese medicines have been increasingly focused on by many studies [7, 8]. Traditional Chinese medicines have been identified as an effective strategy for inflammation intervention, and some herbs have also been found to have a pharmacological effect on anti-inflammation [9]. At present, some prescriptions of traditional Chinese medicines have been used for multiple inflammation treatments [10, 11]. The traditional Chinese medicines have emphasized the symptomatic effect of the prescriptions on the diseases, while the scientific research in cellular and molecular levels on the pharmacological mechanisms of the related prescriptions is lacking [12]. Detoxification II Prescription is one of the traditional Chinese medical strategies for hepatitis treatment and consists capillary artemisia, spreading hedyotis herb, and rhubarb, and those herbs have been confirmed to have some functions in anti-inflammation and improving liver functions [13, 14]. However, the therapeutic effect and pharmacological mechanism remain unclear.

This study attempted to explore the function of Detoxification II Prescription on ACLF and illustrate the regulation mechanism of this traditional Chinese medicine on the inflammation of the liver.

## 2. Materials and Methods

### 2.1. Drug Preparation

The decoction was prepared following Detoxification II Prescription. In brief, 3 g of capillary wormwood herb, 5 g of common peony root, and the powder mixtures including 3 g of spreading hedyotis herb, 1.5 g of Radix Curcumae, and 1.5 g of Rhizoma acori graminei were dissolved by 200 mL of boiled water.

### 2.2. Rat Models

The study was approved by the Medical Ethics Committee, and the culture conditions of the rats followed the guidelines of the National Institute of Health. The Wistar rats, ranging from 6–9 weeks old, were purchased from the Shanghai JAKE biotechnology Co., Ltd. (Shanghai, China), and were housed in a pathogen-free cage at 25°C, 50–70% of relative humidity, and 12 hours dark/light cycle. All rats were provided with filtered tap water and commercial diet ad libitum.

The article "Detoxification II Prescription Suppresses the Th-17/IL-17 Inflammatory Axis to Improve the Liver Function of ACLF-Rats via Inactivating the P38MAPK Pathway" was published in 2021. Journal: J Healthc Eng.

The rats were randomly divided into normal group, ACLF group, and drug intervention group. The rats in ACLF group and drug intervention group were induced by intraperitoneal injection of carbon tetrachloride (2 ml/kg) to form liver cirrhosis and then made into the ACLF-rat models by injecting D-galactosamine (400 mg/kg) and LPS (10 g/kg) intraperitoneally. The rats in drug intervention were irrigated with diluted decoction at 1.5 mL/10g for 21 days, and the rats in ACLF group were treated wtih the normal saline at 1.5 mL/10g for 21 days. Moreover, ACLF rats were treated with SB203580 (S1076; 2 mg/kg/day; Selleck Chemicals, Shanghai, China) for 2 weeks to inhibit the activation of P38MAPK pathway. The flow of experiment is shown in Figure 1.

### 2.3. Flow Cytometry

The percentage of Th-17 cells was detected by flow cytometry assay. The peripheral bloods collected from the rats were treated with NH4Cl lysis solution, to remove the red blood cells. Caltag™ and Fix& Perm® reagents purchased from Thermo Fisher Scientific (Waltham, MA, USA) were used for cell staining. In short, the lymphomononuclear cells isolated from the blood sample of the rats were incubated with fluorochrome-labeled antibodies (anti-CD4, Thermo Fisher Scientific, Waltham, MA, USA) at 5 × 10^5^ cells at 4°C for 30 min, and then, the cells were analyzed by flow cytometry assay.

### 2.4. qRT-PCR

The total RNAs of the tissues or cells were extracted with TRIzol reagent, and the concentration of the extracts were measured by UV spectrophotometry. The total RNAs were retranslated as cDNA by using the TaqMan MicroRNA Reverse Transcription Kit (Applied Biosystems, Foster city, CA). According to the instructions of the KAPA qRT-PCR kit (Sigma-Aldrich, Missouri, USA), the reaction system was prepared for PCR. The reaction conditions included denaturation at 95°C for 3 min, followed by amplification for 40 cycles at 95°C for 12 s, at 60°C for 40 s, and at 70°C for 30 s. The relative expression levels of the related factors were calculated with with the 2^−(ΔΔCt)^ method. The information of the primers is listed in Table 1.

### 2.5. Determination of the Liver Function Indexes

The levels of ALT, AST, TBiL, ALB, and CHE were measured by using the related standard kits purchased from Wuhan Saipei Biotechnology Co., Ltd. (Wuhan, China) according the related instructions.

### 2.6. Western Blot

The Th-17 cells were isolated from the peripheral bloods collected of the rats. The total proteins of Th-17 cells were extracted by RIPA buffer, and then, the concentration of extracts was measured by using the BCA kit under a UV Spectrophotometer. After concentration normalizing, the proteins were separated with sodium dodecyl sulfate polyacrylamide gels and then were translated on the polyvinylidene fluoride membranes (Bio-Rad, CA, USA) by the wet-translation method. After that, the membranes were blocked with 5% fat-free milk for 1 hour and incubated with the related primary antibodies overnight. Subsequently, the membranes were washed with TBST (3 × 15 min) and then were incubated with second membranes for 2 hours. Finally, the membranes were washed with TBST (3 × 10 min) and then observed by using a chemiluminescence detection system, and the relative concentration of the factors was calculated. p-P38 (1 : 1000, AB_2835330) was from Thermo Fisher, Massachusetts, USA; *β*-actin (1 : 1000) was from Thermo Fisher, Massachusetts, USA.

The article "Detoxification II Prescription Suppresses the Th-17/IL-17 Inflammatory Axis to Improve the Liver Function of ACLF-Rats via Inactivating the P38MAPK Pathway" was published in 2021. Journal: J Healthc Eng.

### 2.7. Data Analysis

The experiments in this study were performed three times, independently. The data were analyzed by the chi-squared test or ANOVA with Tukey's post hoc test in SPSS 20.0, and the figures were charted with Graphpad Prism 8.0. Moreover, *P* < 0.05 meant that the data in the two groups were statistically significant.

## 3. Results

### 3.1. Detoxification II Prescription Improved the Liver Function of the ACLF-Rats

To investigate the therapeutic effects of Detoxification II Prescription on ACLF, the ACLF-rats in the intervention group were treated with Detoxification II Prescription, and the rats in the control group were treated with the intervention of physiological saline. Moreover, the levels of ALT, AST, TBiL, CHE, and ALB in the serums of the rats were observed by using the related standard kits. It was found that the rats treated with Detoxification II Prescription expressed low ALT, AST, and TBiLs levels compared with the ACLF-rats treated with placebos (Figure 2, *P* < 0.05). Besides, the study also found that the levels of CHE and ALB increased significantly in the ACLF-rats treated with Detoxification II Prescription compared with the ACLF-rats treated with the normal saline. Those observations suggested that Detoxification II Prescription could effectively improve the symptoms of ACFL (Figure 2, *P* < 0.05).

### 3.2. Detoxification II Prescription Regulated the Levels of Th-17 and IL-17

To delve the regulation mechanism of Detoxification II Prescription on liver failure, the levels of IL-17 IL-6, and IFN-*γ* in the serums and the percentage of Th-17 in CD4 cells of the rats were also observed by flow cytometry assay and western blot, respectively. The results showed that the Th-17 and IL-17 levels were significantly upregulated in the rats treated with the decoction compared with the rats treated with placebo (Figure 3, *P* < 0.05). Moreover, it was also observed that the levels of IL-6 and IFN-*γ* in the serums of the ACLF-rats significantly decreased after the treatment of Detoxification II Prescription (Figure 3, *P* < 0.05). Those observations suggested that Detoxification II Prescription could improve the inflammation of the ACLF-rats and promote the expression of Th-17 and IL-17.

The article "Detoxification II Prescription Suppresses the Th-17/IL-17 Inflammatory Axis to Improve the Liver Function of ACLF-Rats via Inactivating the P38MAPK Pathway" was published in 2021. Journal: J Healthc Eng.

### 3.3. Detoxification II Prescription Induced p38MAPK Inactivation in Liver Cells of ACLF-Rats

To reveal the functional mechanism of Detoxification II Prescription on ACLF, the liver tissues of the rats were obtained, and western blot was used to observe the activity of the p38MAPK pathway in the liver cells. The results reflected that the expression levels of p-P38 were extremely downregulated in the tissues of decoction-treated rats compared with those of placebo-treated rats (Figure 4. *P* < 0.05). These observations suggested that Detoxification II Prescription could inhibit the activity of the p38MAPK pathway in the improvement of liver failure.

### 3.4. P38MAPK Downregulation Improved the Liver Function Indexes of the ACFL-Rats

The verify the role of P38MAPK in the progression of ACLF, the ACFL-rats were treated with P38MAPK inhibitor (SB203580) lentivirus carrier, and the liver function indexes of the ACLF-rats including the levels of ALT, AST, TBiL, CHE, and ALB were measured. The results showed that P38MAPK downregulation remarkably inhibited the expression level of P38MAPK, and P38MAPK downregulation effectively reduced the levels of ALT, AST, and TBiL and improved the levels of CHE and ALB in the serums of the ACLF-rats (Figure 5, *P* < 0.05). These observations suggested that the P38MAPK pathway played an important role in the progression of ACLF.

### 3.5. P38MAPK Downregulation Decreased the Levels of Th-17 and IL-17

To delve whether Detoxification II Prescription regulates the level of the Th-17/IL-17 inflammatory axis via the p38MAPK pathway, the rats were injected with sh-P38 lentivirus carrier, and the levels of Th-17 and IL-17 were observed in the serums of the rats. The results showed that the downregulated p38MAPK effectively reduced the ratio of Th-17 cells in CD4^+^ cells and suppressed the expression of IL-17 in the serums of the ACLF-rats (Figure 6, *P* < 0.05). These observations suggested that Detoxification II Prescription could suppress the activation of the Th-17/IL-17 axis to improve the ACLF via inactivating the p38MAPK pathway.

## 4. Discussion

Currently, liver failure remains an intractable disease which takes a great challenge on the medical system in the world, and ACLF treatment has became a challenge of model medicine [14]. At present, increasing studies have revealed the protective effects of traditional Chinese medicines on the liver, and several studies have indicated that some decoction processed according to the related prescription of traditional Chinese medicines could effectively improved the symptoms of liver-related diseases such as liver failure and hepatic sclerosis [15, 16]. In this study, the effects of Detoxification II Prescription on liver failure have been explored, and the pharmacological mechanism of Detoxification II Prescription were also illustrated via verifying in the rat model.

The article "Detoxification II Prescription Suppresses the Th-17/IL-17 Inflammatory Axis to Improve the Liver Function of ACLF-Rats via Inactivating the P38MAPK Pathway" was published in 2021. Journal: J Healthc Eng.

ACLF-rats are always used for the research of acute-on-chronic liver failure [17]. The levels of ALT, AST, TBiL, ALB, and CHE have been widely used as the physiological indexes for the diagnosis of the liver-related diseases in clinic [18]. To investigate the effect of Detoxification II Prescription on ACLF, the ACLF models were also treated with GaIN to establish the ACLF-rats, and it was found that the levels of ALT, AST, and TBiL in the serums of the ACLF-rats increased, while the levels of ALB and CHE significantly decreased compared with normal rats. Moreover, the results of this study supported that the ACLF-rats treated with the decoction processed according to Detoxification II Prescription expressed low IL-17, IL-6, and IFN-*γ*, which suggested that detoxification II Prescription could effectively reduce inflammatory levels and improve the liver injury of ACLF-rats. Following the instruction Detoxification II Prescription, the capillary artemisia, spreading hedyotis herb, and rhubarb were boiled to obtain the decoction, and the compounds in herbs were absorbed and then influenced the internal environments of the patients' bodies. It was found that Detoxification II Prescription obviously decreased the levels of inflammatory factors and improved the levels of ALT, AST, TBiL, ALB, and CHE of ACLF-rats, which supported the therapeutic effect of Detoxification II Prescription on ACLF treatment. The study has proved that Yinchen Wuling Power, one of the traditional Chinese medicines, could effectively improve the jaundice hepatitis, liver fibrosis, hyperlipidemia, and early diabetes, and Yinchen plays an important role in this prescription [19]. *Hedyotis diffusa* serves as an inhibitor which could effectively restrain the malignant progression of the tumor, and the recent study has indicated that the decoction of *Hedyotis diffusa* could improve the acute liver injury of rats induced by LPS [20]. Besides, rhubarb is also a major component of the Detoxification II Prescription, and several studies have indicated that proper rhubarb plays a protector role in preventing the hepatic inflammation induced by alcohol or virus infection [13]. Those proofs support the curative effect of Detoxification II Prescription on ACLF.

The article "Detoxification II Prescription Suppresses the Th-17/IL-17 Inflammatory Axis to Improve the Liver Function of ACLF-Rats via Inactivating the P38MAPK Pathway" was published in 2021. Journal: J Healthc Eng.

The level of Th-17 cells is an important biomarker which could directly reflect the inflammatory level of the patients, and increased level of Th-17 cells has been observed in the serums of the patients with ACLF [21]. In this study, it was also found that the ratio of IL-17-positive CD4^+^ cells was significantly upregulated in the serums of ACLF cells. Moreover, this study also verified that the ratio of IL-17-positive CD4 in serum of the ACLF-rats accepted the intervention of Detoxification II Prescription was significantly downregulated compared with the ACLF-rats treated with placebo. Besides, multiple studies have confirmed that IL-17 excreted by Th-17 cells involves the progression of chronic hepatitis, and increased IL-17 level could aggravate the symptom of liver failure [22, 23]. The study has also proved that the dysfunctions of Th-17/IL-17 inflammatory axis play a key role in the progression of chronic hepatitis induced by HBV and HCV [24]. Thus, this study suggested that Detoxification II Prescription could alleviate the symptom of ACLF.

Furthermore, the activated p38MAPK pathway was observed in the ACLF-rats in this study, and the rats with intervention of Detoxification II Prescription expressed low p38MAPK activity. Aberrant activation of p38MAPK is related with the several inflammations. Several studies have indicated that hepatitis B could promote the accumulation of antiapoptotic protein and then induce hepatocellular carcinoma cells survive via activating the p38MAPK pathway [25]. Moreover, it has been confirmed that the p38MAPK pathway is related with the differentiation of Th-17 cells [26]. This study also proved that the inactivated p38MAPK pathway could effectively reduce the expression level of IL-17. Therefore, this study supported that Detoxification II Prescription could visibly inhibit the activation of Th-17/IL-17 inflammatory via inactivating the p38MAPK pathway.

In conclusion, this study confirmed that Detoxification II Prescription could effectively improve the symptoms of ACLF-rats and illustrated that Detoxification II Prescription could inhibit the Th-17/IL-17 inflammatory axis via inactivating the p38 MAPK pathway.

## Figures and Tables

**Figure 1:** The flowchart of the study.

**Figure 2:** Detoxification II Prescription improved the liver functions of the ACLF-rats. (a–e) The levels of ALT, AST, TBiL, ALB, and CHE in the serums of the rats were measured by using the related kits. ^*∗*^*P* < 0.05.

The article "Detoxification II Prescription Suppresses the Th-17/IL-17 Inflammatory Axis to Improve the Liver Function of ACLF-Rats via Inactivating the P38MAPK Pathway" was published in 2021. Journal: J Healthc Eng.

**Figure 3:** Detoxification II Prescription improved the inflammatory levels of the ACLF-rats. (a-b) The percentages of Th-17 cells in CD4^+^ cells of the rats were measured by flow cytometry assay. (c–e) The relative levels of IL-17, IL-6, and INF-*γ* were measured by qRT-PCR.

**Figure 4:** Detoxification II Prescription inhibited the P38MAPK in liver tissues of the rats. (a-b) The relative expression level of P38MAPK in the liver tissues of the rats was measured by western blot. ^*∗*^*P* < 0.05.

**Figure 5:** P38MAPK downregulation improved the liver functions of the ACLF-rats. (a–e) The levels of ALT, AST, TBiL, ALB, and CHE in the serums of the rats were measured by using the related kits. ^*∗*^*P* < 0.05.

**Figure 6:** P38MAPK downregulation improved the inflammatory levels of the ACLF-rats. (a-b) The percentages of Th-17 cells in CD4^+^ cells of the rats were measured by flow cytometry assay. (c–e) The relative levels of IL-17, IL-6, and INF-*γ* were measured by qRT-PCR.

**Table 1:** The information of the primers.

Name of the primer	Sequences
IL-6-F	5′-TGCTCCTGGTGTTGCCTGCT-3′
IL-6-R	5′-AGCCACTGGTTCTGTGCCTGC-3′
IL-17-F	5′-ACCAATCCCAAAAGGTCCTC-3′
IL-17-R	5′-GGGGACAGAGTTCATGTGGT-3′
IFN-*γ*-F	5′-GCATCCAAAAGAGTGTGGAG-3′
IFN-*γ*-R	5′-GCAGGCAGGACAACCATTAC-3′
U6-F	5′-CTCGCTTCGGCAGCACA-3′
U6-R	5′-AACGCTTCACGAATTTGCGT-3′

## Data Availability

Data to support the findings of this study are available on reasonable request from the corresponding author.
